The article "Correlation of Complex Impacted Mandibular Teeth with Pericoronitis and Effect of Minimally Invasive Tooth Extraction on Patients' Long-term Outcome of Masticatory Ability" was retracted in 2023. Reasons: signs of a paper mill; suspected computer-generated content; unreliable results or conclusions; lack of ethics approval or compliance.

# Correlation of Complex Impacted Mandibular Teeth with Pericoronitis and Effect of Minimally Invasive Tooth Extraction on Patients' Long-term Outcome of Masticatory Ability

**DOI:** 10.1155/2022/6389900

**Published:** 2022-10-17

**Authors:** Tinghong Nie, Bojie Chang, Lili Tian, Shansong Cao, Junjie Wang, Haitao Qi, Lirong Gao

**Affiliations:** Department of Stomotology, Tianjin Baodi Hospital/Baodi Clinical College of Tianjin Medical University, Tianjin 301800, China

## Abstract

**Objective:**

To explore the correlation of complex impacted mandibular teeth and pericoronitis, as well as the effect of minimally invasive tooth extraction on patients' long-term outcomes of masticatory ability.

**Methods:**

A total of 101 patients with complex impacted teeth who were treated in our hospital from March 2019 to June 2021 were selected and divided into the control group (*n* = 55) and the observation group (*n* = 46) according to the different treatment methods. The patients in the control group were given conventional extraction treatment, and the patients in the observation group were given minimally invasive extraction treatment. The clinicopathological features of patients complicated by pericoronitis were observed and the relationship between complex impacted mandibular teeth and pericoronitis was discussed. Additionally, we made statistics on operative time (OT), intraoperative blood loss (IBL), dental socket integrity score, and adverse reactions (ARs) and compared the clinical efficacy between the observation group and control group. The Visual Analogue Scale (VAS) and Oral Health Impact Profile scale (OHIP-14) were utilized for pain assessment and oral health status evaluation, respectively. Bite force (BF) and masticatory efficiency were also measured.

**Results:**

OG showed less OT and IBL than CG, with a higher dental socket integrity score (*P* < 0.05). In addition, OG outperformed CG with a higher overall response rate and a lower incidence of ARs (*P* < 0.05). The pretreatment VAS score, mouth-opening degree, and OHIP-14 score differed insignificantly between groups (*P* > 0.05). After treatment, the VAS score of OG decreased, while the mouth-opening degree and OHIP-14 score increased (*P* < 0.05). Finally, the mastication ability was higher in OG at 7 days postoperatively, but there was no difference between groups at 6 months postoperatively (*P* > 0.05).

**Conclusion:**

Complex mandibular impacted teeth can easily induce pericoronitis, so clinicians should pay attention to the influencing factors of pericoronitis. Minimally invasive surgery for complex impacted mandibular teeth can effectively improve treatment outcomes, accelerate patient rehabilitation, and provide more effective protection for patients' oral health and masticatory ability, which is worth promoting in clinical use.

The article "Correlation of Complex Impacted Mandibular Teeth with Pericoronitis and Effect of Minimally Invasive Tooth Extraction on Patients' Long-term Outcome of Masticatory Ability" was retracted in 2023. Reasons: signs of a paper mill; suspected computer-generated content; unreliable results or conclusions; lack of ethics approval or compliance.

## 1. Introduction

Teeth that cannot erupt into the normal occlusal position due to their improper position in the jawbone are called impacted teeth [1]. According to the investigation, more than 20% of adults have impacted teeth to varying degrees, and the prevalence is constantly on the rise [2]. Impacted teeth are mostly found in the mandibular and maxillary third molars, among which complex mandibular impacted teeth are the most common, accounting for approximately 60-70% of all impacted teeth [3]. The most typical clinical symptom of complex impacted mandibular teeth is obvious intermittent toothache or gingival swelling, accompanied by a great risk of infection, which is easy to induce pericoronitis or periodontitis [4]. In addition, if the patient suffers from complications and misses the best treatment time, it will probably lead to a large area of jaw necrosis, jaw cyst lesions, and even oral cancer, which will endanger the life safety of the patient [5]. At present, extraction is still the mainstay of treatment for complex impacted mandibular teeth in clinic. Although the operation is not difficult and the success rate is relatively high, the incidence of postoperative wound pain and diffuse inflammation is high, which is the key problem affecting the prognosis and recovery of patients [6, 7].

With consistent development and improvement, minimally invasive techniques have contributed to extremely remarkable application results in the medical field. For instance, laparoscopic surgery and stone surgery based on minimally invasive techniques have been shown to be more effective and safer than traditional surgical modalities [8–10]. In the treatment of impacted mandibular teeth, minimally invasive surgery has gradually obtained clinical recognition and become one of the preferred treatment options for patients [11]. Currently, minimally invasive techniques like high-speed turbine technology have been proved to have excellent application effects in dental implants and orthodontic treatment [12, 13], but the research concerning its application in complex impacted mandibular teeth is still rare.

Accordingly, this study will carry out correlation analysis on the correlation of complex impacted mandibular teeth with pericoronitis and discuss the application effect of minimally invasive tooth extraction, so as to provide novel evidence for future clinical treatment of such patients and improve patient safety.

## 2. Materials and Methods

### 2.1. Patient Data

A total of 101 patients with complex impacted mandibular teeth who were treated in our hospital from March 2019 to June 2021 were selected and divided into the control group (*n* = 55) and the observation group (*n* = 46) according to the different treatment methods. Besides, in order to understand the correlation between complex impacted mandibular teeth and pericoronitis, the patients with impacted mandibular teeth complicated with pericoronitis were set as group A (*n* = 31), and the patients with impacted mandibular teeth without pericoronitis were set as group B (*n* = 70).

The article "Correlation of Complex Impacted Mandibular Teeth with Pericoronitis and Effect of Minimally Invasive Tooth Extraction on Patients' Long-term Outcome of Masticatory Ability" was retracted in 2023. Reasons: signs of a paper mill; suspected computer-generated content; unreliable results or conclusions; lack of ethics approval or compliance.

### 2.2. Inclusion and Exclusion Criteria

Inclusion criteria are as follows: patient's age >18 years; the patient was diagnosed with a complex impacted mandibular tooth and confirmed by X-rays and underwent extraction treatment in our hospital; patient himself/herself signs an informed consent form; and patient data are complete.

Exclusion criteria are as follows: patients with mental, cognitive, and communication disorders; patients with low treatment compliance; patients with periodontitis, caries, and other dental conditions; and patients with blood or immune diseases.

### 2.3. Methods

After admission, both groups received routine X-ray examination to explore the correlation of impacted mandibular teeth with adjacent tissues. After disinfection, 3 mL lidocaine hydrochloride injection (Shanghai Zhaohui Pharmaceutical, SFDA Approval No. H31021072) was used for block anesthesia of the inferior alveolar nerve, and an incision was made at the buccal gum to fully expose the bone overlying the impacted mandibular tooth crown. Subsequently, patients in the control group were treated with bone chisel for conventional extraction: following the opening of the mucoperiosteal flap with a gingival separator, bone removal was performed using bone chisel, and the resistance of the crown root was relieved after enlarging the gap. After the impacted tooth became loose, the root crown was removed with ultrasonic osteotome, the alveolar fossa was cleaned, and the wound was fully washed with 0.9% sodium chloride injection before suturing. Observation group was treated with minimally invasive plus high-speed turbine tooth extraction: the alveolar bone at the alveolar site and the top of the alveolar bone was ground off according to the patient's oral condition, and the crown was exposed (bone grinding is not required if the area of the patient's bone window is too large). Separation was then performed several times, using the patient's alveolar crest as the surgical approach. After all the resistance was removed, a turbine was used for root division and complete extraction of the complete dental tissue.

### 2.4. Efficacy Evaluation

Marked response: the patient's symptoms disappeared completely and the masticatory function returned to normal. Response: the patients' symptoms basically disappeared and the masticatory function recovered to a certain extent. Nonresponse: no change in symptoms nor recovery of masticatory function. Overall response rate (ORR) = (marked response cases + response cases)/Total number of cases × 100% [14].

The article "Correlation of Complex Impacted Mandibular Teeth with Pericoronitis and Effect of Minimally Invasive Tooth Extraction on Patients' Long-term Outcome of Masticatory Ability" was retracted in 2023. Reasons: signs of a paper mill; suspected computer-generated content; unreliable results or conclusions; lack of ethics approval or compliance.

### 2.5. Follow-up for Prognosis

All patients were followed up for 6 months after discharge, with either outpatient or telephone questioning each month to observe their recovery.

### 2.6. Endpoints

(1) The incidence of pericoronitis in patients with complex impacted mandibular teeth was counted. (2) Operation condition: the operative time (OT), intraoperative blood loss (IBL), and dental socket integrity score of both cohorts were counted [15]. (3) Safety: the adverse reactions (ARs) of patients from postoperative to discharge were recorded to calculate the incidence of ARs. (4) Clinical efficacy. (5) Pain and mouth-opening degree: pain assessment, which was made using the Visual Analogue scale (VAS), was performed before and 2 d after surgery. VAS score can better indicate the severity of pain and the degree of pain relief before and after treatment. Among them, 0 point means no pain, 1-3 points means mild pain, 4-6 points means moderate pain, and 7-10 points means severe pain. (6) Oral health status: oral health evaluation was performed using the Oral Health Impact Profile scale (OHIP-14) [16]. OHIP-14 provided oral health assessment to patients from four dimensions of functional limitation, physical disability, physical pain, and social disability, with a total score of 10 points. A lower score indicates a better oral health condition for the patient. (7) Masticatory ability: the occlusal force tester measured the maximum bite force (BF) of patients. The patient was asked to chew 2.0 g peanuts 20 times on the left and right sides. The chews were then collected and mixed with double distilled water to a volume of 1000 mL. After stirring the middle and upper suspension for 1 min, a spectrophotometer was used to determine the absorbance value as the patient's mastication efficiency. The test was carried out 7 days postoperatively and 6 months after prognosis.

### 2.7. Statistics and Methods

SPSS22.0 performed statistical analysis, and statistical significance was indicated by *P* < 0.05. The Chi-square test was used for comparisons of count data (*n* (%)), and the independent sample *t*-test and paired *t*-test were used for comparisons of measurement data ($\bar{\chi }$ ± *s*).

## 3. Results

### 3.1. Incidence of Pericoronitis in Patients with Complex Impacted Mandibular Teeth

The intergroup comparison of patients' clinicopathological data revealed no notable difference in age and sex between groups (*P* > 0.05); however, group A had more cases of pericoronal blind pocket depth ≥3 mm, sleep insufficiency, no physical exercise, brushing times <1/d, and family medical history than group B (*P* < 0.05). As shown in Table 1, it can be seen that when the abovementioned conditions exist in patients with complex impacted mandibular teeth, clinical attention should be paid to prevent the occurrence of pericoronitis.

The article "Correlation of Complex Impacted Mandibular Teeth with Pericoronitis and Effect of Minimally Invasive Tooth Extraction on Patients' Long-term Outcome of Masticatory Ability" was retracted in 2023. Reasons: signs of a paper mill; suspected computer-generated content; unreliable results or conclusions; lack of ethics approval or compliance.

### 3.2. Comparison of Clinical Data

Then, to ensure the comparability of the results of the two treatment methods, we compared the data of observation group and control group again. The two groups differed insignificantly in various data (*P* > 0.05), confirming the credibility of the experimental results, as shown in Table 2.

### 3.3. Comparison of Operation Conditions

As shown in Figure 1, the observation group had less OT and IBL than the control group (*P* < 0.05). The comparison of dental socket integrity scores revealed a higher score in the observation group compared than the control group (*P* < 0.05).

### 3.4. Comparison of Clinical Efficacy

See Table 3 for efficacy of both cohorts of patients. In the observation group, marked response and response were found in 41.3% and 50.0% patients, respectively, while those with nonresponse accounted for 8.7% only, with an ORR of 91.30% that was higher than the control group (*P* < 0.05).

### 3.5. Comparison of Safety

As shown in Table 4, the incidence of ARs in the observation group was 8.7% versus 23.6% in the control group. The data revealed a lower incidence of ARs in the observation group versus the control group (*P* < 0.05).

### 3.6. Comparison of Pain and Mouth-Opening

As shown in Figure 2, the two cohorts were nonsignificantly different in pretreatment VAS score and mouth-opening degree (*P* > 0.05). In the control group, the VAS score on day 2 after treatment was similar to the baseline (before treatment) (*P* > 0.05), but the VAS score of the observation group decreased on the 2nd day after treatment versus the baseline and control group (*P* < 0.05). Both groups showed a wider mouth-opening degree than the baseline, especially in the observation group (*P* < 0.05).

### 3.7. Comparison of Oral Health Status

The OHIP-14 score results shown in Figure 3 demonstrated no difference between groups prior to treatment (*P* > 0.05). While the post-treatment functional limitation, physiological disability, physical pain, and social disability scores were even lower in the observation group than the control group (*P* < 0.05). In both groups, a decreased OHIP-14 score was observed after treatment (*P* < 0.05).

The article "Correlation of Complex Impacted Mandibular Teeth with Pericoronitis and Effect of Minimally Invasive Tooth Extraction on Patients' Long-term Outcome of Masticatory Ability" was retracted in 2023. Reasons: signs of a paper mill; suspected computer-generated content; unreliable results or conclusions; lack of ethics approval or compliance.

### 3.8. Comparison of Masticatory Ability

As shown in Figure 4, the intergroup comparison of masticatory ability showed better BF and masticatory efficiency in the observation group than the control group at 7 days after surgery (*P* < 0.05). At 6 months postoperatively, markedly enhanced masticatory ability was determined in both cohorts compared with the baseline (*P* < 0.05), but with no statistical intergroup difference (*P* > 0.05).

## 4. Discussion

With the continuous improvement of the technical level of stomatology in China, minimally invasive tooth extraction has gradually been extensively used in stomatology [17]. The complex impacted mandibular tooth is located in a special position in the patient's oral cavity, which is closely combined with the surrounding teeth and affected by narrow oral position, resulting in limited operation space for tooth extraction. In addition, many complicated surgical instruments are involved in the operation of complicated mandibular impacted teeth, which can easily lead to the fracture of surrounding teeth or collision infection, so the extraction of complex impacted mandibular teeth is a difficult and complicated process [18, 19]. Therefore, it is urgent to explore the specific advantages of minimally invasive tooth extraction in clinical practice and promote its application in stomatology.

In this study, we first analyzed the correlation of complex impacted mandibular teeth with pericoronitis. The results showed that a higher percentage of pericoronitis patients had pericoronal blind pocket depth ≥3 mm, sleep insufficiency, no physical exercise, brushing teeth <1/d, and family history, which was also in line with previous studies on the pathological manifestations of pericoronitis [20, 21], indicating that patients with complex impacted mandibular teeth should pay attention to the above situation to prevent the occurrence of pericoronitis. Second, we compared the effects of minimally invasive surgery and traditional surgery in the treatment of complex impacted mandibular teeth. The results determined that the OT and IBL of patients in the observation group were reduced compared with the control group, while the dental socket integrity and clinical efficacy were increased, indicating that minimally invasive surgery was more effective in treating complex impacted mandibular teeth. In previous studies [22, 23], there is evidence that minimally invasive oral surgery is more effective for sialolithiasis and parotid calculi than traditional extractions, which is also consistent with our experimental results. As we all know, traditional tooth extraction for complex impacted mandibular teeth often involves violent percussion, chopping, chiseling, and other harmful operations, which will not only cause serious damage to patients' periodontal tissues but also cause great psychological pressure [24]. In addition, traditional tooth extraction is also susceptible to the influence of factors such as the doctor's skill and the force applied, resulting in inadequate safety of surgical outcomes. Furthermore, during extraction and treatment of complex impacted mandibular teeth, the size, position, number and length of nerves involved, and other factors will affect the operation difficulty [25]. Moreover, violent operation in surgery will further lead to adverse consequences such as postoperative bleeding and wound infection and increase the difficulty of postoperative rehabilitation and the fear of tooth extraction, which is more obvious in traditional tooth extraction [26]. In minimally invasive surgery, complex impacted mandibular teeth can be extracted on the basis of minimal wound, without causing serious pain. At the same time, minimally invasive tooth extraction uses turbines instead of traditional large and bulky surgical instruments, which can fully shorten the OT and reduce the amount of IBL [27]. What's more, the advanced surgical instruments used in minimally invasive tooth extraction have high precision, which can prevent the wound from being infected by bacteria. Meanwhile, the surgical approach that adheres to the periodontal tissue can completely and comprehensively extract complex impacted mandibular teeth, contributing to a lower probability of postoperative ARs [28]. This can be confirmed by lower incidence of postoperative ARs and VAS scores as well as wilder mouth-opening degree in the observation group. And with the improvement of the treatment effect, the overall oral quality of patients is also improved, which explains a higher OHIP-14 score in the observation group versus the control group, demonstrating the excellent application value of minimally invasive surgery for complex impacted mandibular teeth. The chewing ability of patients after tooth extraction is the key that directly affects their normal life and deserves clinical attention. Therefore, in this study, we also explored the effects of the two treatments on the chewing ability of patients [29]. The results determined higher BF and mastication efficiency in the observation group compared with the control group at 7 days after operation, indicating better mastication ability of the observation group at this time. However, there was no difference in chewing ability between the two groups at 6 months after surgery, which might be due to the fact that the patient's oral condition had completely recovered by that time. However, the application of minimally invasive surgery can more effectively ensure the stability of the early postoperative chewing ability of patients and improve the quality of life of patients after surgery, showing that minimally invasive tooth extraction has better clinical value.

The article "Correlation of Complex Impacted Mandibular Teeth with Pericoronitis and Effect of Minimally Invasive Tooth Extraction on Patients' Long-term Outcome of Masticatory Ability" was retracted in 2023. Reasons: signs of a paper mill; suspected computer-generated content; unreliable results or conclusions; lack of ethics approval or compliance.

However, due to the short time frame, we have not been able to assess the long-term oral outcome of patients. Besides, this study is a retrospective analysis, which may have the chance of statistical calculation, so follow-up randomized controlled trials should be carried out as soon as possible for confirmation. Finally, the clinical effect may be affected by the professional skills of clinicians because of the high operative difficulty of minimally invasive surgery in the treatment of complex impacted mandibular teeth, which is also the focus of further exploration.

Conclusively, complex impacted mandibular teeth can easily induce pericoronitis, so patients need to pay attention to the possible influencing factors. Minimally invasive surgery for complex impacted mandibular teeth can effectively improve treatment outcomes, accelerate patient rehabilitation, and provide more effective protection for patients' oral health and masticatory ability, which is worth promoting in clinical use.

## Figures and Tables

**Figure 1:** Comparison of operation conditions. (a) Comparison of operative time between the research group and control group; (b) comparison of intraoperative blood loss between the research group and control group and; (c) comparison of dental socket integrity scores between the research group and control group. Note. ^*∗*^indicates that the difference between the two groups is statistically significant (*P* < 0.05).

**Figure 2:** Comparison of pain and mouth opening. (a) Comparison of VAS score. (b) Comparison of mouth-opening degree. Note. ^#^indicates that the difference is statistically significant compared with that before treatment (*P* < 0.05), and & indicates that the difference is statistically significant compared with the control group (*P* < 0.05).

**Figure 3:** Comparison of oral health status. (a) Comparison of functional limitation scores between the research group and control group. (b) Comparison of physiological disability scores between the research group and control group. (c) Comparison of physical pain scores between the research group and control group. (d) Comparison of social disability scores between the research group and control group. Note. ^#^indicates that the difference is statistically significant compared with that before treatment (*P* < 0.05), and & indicates that the difference is statistically significant compared with the control group (*P* < 0.05).

The article "Correlation of Complex Impacted Mandibular Teeth with Pericoronitis and Effect of Minimally Invasive Tooth Extraction on Patients' Long-term Outcome of Masticatory Ability" was retracted in 2023. Reasons: signs of a paper mill; suspected computer-generated content; unreliable results or conclusions; lack of ethics approval or compliance.

**Figure 4:** Comparison of masticatory ability. (a) Comparison of bite force between the research group and control group. (b) Comparison of masticatory efficiency between the research group and control group. Note. ^#^indicates that the difference is statistically significant compared with that before treatment (*P* < 0.05), and & indicates that the difference is statistically significant compared with the control group (*P* < 0.05).

**Table 1:** Incidence of pericoronitis in patients with complex impacted mandibular teeth.

Indicator	Group A (*n* = 31)	Group B (*n* = 70)	*t*/*χ*^2^	*P*
Age	24.3 ± 6.3	23.6 ± 6.3	0.517	0.606

Pericoronal blind pocket depth			13.690	<0.001
<3 mm	26 (83.9)	30 (42.9)		
≥3 mm	5 (16.1)	40 (57.1)		

Sex			0.046	0.829
Male	16 (51.6)	35 (50.0)		
Female	15 (48.4)	35 (50.0)		

Sleep situation			8.748	0.003
<8 h	7 (22.6)	39 (55.7)		
≥8 h	24 (77.4)	31 (44.3)		

Brushing times			10.420	0.001
<1 time/d	13 (41.9)	54 (77.1)		
≥1 time/d	18 (58.1)	16 (22.9)		

Physical exercise			7.443	0.006
Yes	9 (29.0)	40 (57.1)		
No	22 (71.0)	30 (42.9)		

Family medical history			13.330	<0.001
Yes	14 (45.2)	9 (12.9)		
No	17 (54.8)	61 (87.1)		

**Table 2:** Comparison of clinical data.

Indicator	Control group (*n* = 55)	Observation group (*n* = 46)	*t*/*χ*^2^	*P*
Age	24.9 ± 6.9	23.1 ± 5.5	1.429	0.156

Pericoronal blind pocket depth			0.327	0.567
<3 mm	30 (54.5)	26 (56.5)		
≥3 mm	25 (45.5)	20 (43.5)		

Sex			0.241	0.624
Male	29 (52.7)	22 (47.8)		
Female	26 (47.3)	24 (52.2)		

Sleep situation			0.676	0.411
<8 h	27 (49.1)	19 (41.3)		
≥8 h	28 (50.9)	27 (58.7)		

Brushing times			0.047	0.828
<1 time/d	35 (63.6)	32 (69.6)		
≥1 time/d	20 (36.4)	14 (30.4)		

Physical exercise			0.241	0.624
Yes	29 (52.7)	20 (43.5)		
No	26 (47.3)	26 (56.5)		

Family medical history			0.528	0.468
Yes	11 (20.0)	12 (26.1)		
No	44 (80.0)	34 (73.9)		

Pericoronitis			0.018	0.893
Yes	15 (27.3)	16 (34.8)		
No	40 (72.7)	30 (65.2)		

**Table 3:** Comparison of clinical efficacy.

Group	Marked response	Response	Nonresponse	ORR (%)
Control group (*n* = 55)	18 (32.7)	23 (41.8)	14 (25.5)	74.5
Observation group (*n* = 46)	19 (41.3)	23 (50.0)	4 (8.7)	91.30
*χ * ^2^				4.804
*P*				0.028

**Table 4:** Comparison of safety.

Group	Lower jaw pain	Wound infection	Wound swelling	Restricted mouth movement	ARs (%)
Control group (*n* = 55)	5 (9.1)	2 (3.6)	4 (7.3)	2 (3.6)	13 (23.6)
Observation group (*n* = 46)	2 (4.3)	0 (0.0)	1 (2.2)	1 (2.2)	4 (8.7)
*χ * ^2^					3.994
*P*					0.046

## Data Availability

The raw data supporting the conclusion of this article will be available by the authors without undue reservation.
